# The Elevated Circ_0067835 Could Accelerate Cell Proliferation and Metastasis via miR-1236-3p/Twist2 Axis in Hepatocellular Carcinoma

**DOI:** 10.1155/2022/2825172

**Published:** 2022-10-10

**Authors:** Jianghong Chen, Zihan Qi

**Affiliations:** ^1^Department of General Surgery, Tranditional Chinese Medicine Hospital of Chongqing Jiulongpo Area, Chongqing 400060, China; ^2^Department of Animal and Plant Quarantine, Hebei Agricultural University, Baoding 071001, China

## Abstract

Hepatocellular carcinoma (HCC) is a malignant cancer with leading mortality worldwide. Circ_0067835 is a circRNA which plays an important role in various kinds of tumor, while the potential functions of circ_0067835 in HCC remains unclear. In this study, our results of microarray and real-time PCR (RT-PCR) showed that it was obviously elevated in human HCC tumor tissues and HCC cell lines. Inhibition of circ_0067835 restrained cell proliferation and migration in vitro. Furthermore, miR-1236-3p was decreased in tumor samples, and it was indicated to be a target of circ_0067835. Moreover, Twist2 was established to be elevated in HCC tissues, and we identified it as the direct target of miR-1236-3p. Finally, we found that knockdown of miR-1236-3p could reverse the circ_0067835 inhibition effects in HCC cells. In conclusion, our study demonstrated that circ_0067835 contributed to promoting hepatocellular carcinoma cell proliferation and metastasis through downregulating miR-1236-3p expression and then elevating Twist2 expression, which might provide a new vision for HCC patients.

## 1. Introduction

HCC has been regarded as a common cancer in the world, and it owns the second highest mortality, moreover, it is a leading cause for human cancer-related death of the world [1–3]. About 30% HCC patients are diagnosed at early stages and receive curative treatments, such as liver resection, chemotherapy, radiation therapy, etc. [2–5]. However, many HCC patients are diagnosed at later stages, which shows a poor prognosis for them [2–5]. Thus, it is urgently essential to find some diagnostic markers to make earlier diagnoses and identify therapeutic targets to improve the clinical efficacy for HCC patients.

Circular RNAs (circRNAs) are couples of noncoding RNAs; they own the closed-loop structure that have no terminal 5′ caps and 3′ polyadenylated tails [6–9]. circRNAs play crucial roles in the progression of various cancers, including HCC [10–13]. For example, the upregulated circ_001306 could enhance HCC cell growth by regulating miR-584-5p/CDK16 axis [10]. Circ_0067835 is a circRNA plays an important role in some cancers [14, 15]. For example, it could accelerate the malignant development of endometrial cancer via miR-545-3p/FAM98A axis [14]. Furthermore, it has been revealed that circ_0067835 knockdown could suppress cell progression and enhance cell radiosensitivity of colorectal cancer partially by sponging with miR-296-5p/IGF1R axis [15]. But the expression of it in HCC remained unclear. Thus, we wanted to investigate the expression and functions of it in HCC patients.

Researches have revealed that circRNAs can regulate various cell biology through interacting with couples of microRNAs (miRNAs), that has been named as a competing endogenous RNA (ceRNA) mechanism [6–9, 16, 17]. miRNAs may regulate various functions through binding with the 3′ untranslated regions (UTR) of downstream target genes in HCC [18–21]. miR-1236-3p has been demonstrated to be involved with some digestive system cancers, such as gastric cancer [22, 23] and colorectal cancer [24]. However, the functions of miR-1236-3p in HCC also remained unclear. Interestingly, miR-1236-3p has been predicted to be a sponging miRNA of circ_0067835. Thus, we might hypothesize that circ_0067835 might affect the progression and metastasis of HCC through interacting with miR-1236-3p.

The study aims at investigating and verifying this hypothesis to clarify the role of circ_0067835 and miR-1236-3p in HCC cell proliferation and metastasis and identify the new therapeutic target for treating HCC.

## 2. Materials and Methods

### 2.1. Clinical Tissue Samples

56 paired tumor tissues and adjacent nontumor tissues were obtained from HCC patients in our hospital from May 2013 to September 2016, which were stored at -80°C. The clinical characters of HCC patients were listed in Table 1. Among these patients, 29 of them were diagnosed with metastasis, including intrahepatic metastasis, lymph node metastasis, and distant metastasis with target organs, such as lung and bones. This research was approved by Tranditional Chinese Medicine Hospital Ethics Committee of Chongqing Jiulongpo Area (approval number: JLPTCMHWEC2013003; location: No.160 of Longquan Village in Mawang Town, Jiulongpo Area, Chongqing).

### 2.2. Diagnostic Criteria for HCC Patients

The criteria are as follows: (1) 40-80 years old; (2) pathological examination confirmed it; (3) no treatments were given to patients, such as surgery, radiotherapy, chemotherapy, etc.; (4) the informed consent was signed for each subject. The adjacent nontumor tissues were obtained 2 cm away from the tumor tissues.

### 2.3. circRNA Microarray

For performing the microarray analysis, 3 paired of tumor tissues and nontumor tissues were obtained from HCC patients. Then total RNAs were collected from them and were transferred into the fluorescent cRNA by using an Arraystar Super RNA Labeling Kit (Arraystar, USA). Moreover, they were purified by RNeasy Plant Mini Kit (Qiagen, Hilden, Germany). Additionally, the microarray hybridizations on Arraystar Human circRNA Array chip (Agilent, USA) were performed according to its protocol. Finally, it was scanned by an Agilent Scanner (Agilent, Santa Clara, CA, USA), which was analyzed with the Agilent supporting software.

### 2.4. Cell Culture

The human hepatocyte cell line HL-7702 (San Diego, CA, USA) and human HCC cells Hep3B, HepG2, PLC5, and Huh-7 were obtained from American Type Culture Collection (ATCC, USA). HCC cells and hepatocyte cells were, respectively, cultured in DMEM Medium (Invitrogen, USA), which was added with 10% fetal bovine serum (FBS; Gibco, USA), 1% penicillin (Hyclone, USA) and 1% streptomycin (Hyclone, USA). Finally, they were cultured in an environment with the temperature of 37°C and 5% CO_2_.

### 2.5. Construction of siRNA and Cell Transfection

Small interfering RNA (siRNA) for circ_0067835 and the siRNA negative control (si-NC) were obtained from RiBo Biotech (GuangZhou, China), which were subcloned into pcDNA3.1, thereby generating the inhibition vector of circ_0067835 (si-circ_0067835) and its control (si-NC). PLC5 or HepG2 cells were planted on 6-well plates to about the confluence of 60% in each well, then si-circ_0067835 or si-NC (catalogue number: siN0000001-1-5, RiBo Biotech, GuangZhou, China) was, respectively, transfected into the prepared cells with Lipofectamine 2000 (Invitrogen, USA) according to the protocol. Cells were cultured for 24 h before using in subsequent experiments, and cells with circ_0067835 inhibition were obtained. For miRNA transfection assay, cells were prepared on the plates as before, miR-1236-3p mimics (catalogue number: miR10005591-1-5, RiBo Biotech, GuangZhou, China), mimics NC (catalogue number: miR1N0000001-1-5, RiBo Biotech, GuangZhou, China), miR-1236-3p inhibitor (catalogue number: miR20005591-1-5, RiBo Biotech, GuangZhou, China), and inhibitor NC (catalogue number: miR2N0000001-1-5, RiBo Biotech, GuangZhou, China) were, respectively, transfected into the target cells with Lipofectamine 2000 according to its protocol.

### 2.6. RNA Extraction and Quantitative Real-Time PCR

Total RNAs of tissues and cells were extracted with Trizol reagent (Invitrogen, USA) in accordance with its protocol. 1 *μ*g total RNAs were reversed into cDNA by using PrimeScript™ RT reagent Kit (Takara, Beijing, China). PCR primers are showed in Table 2, and the parameters are as follows: 37°C for 15 minutes and 85°C for 5 seconds and keep in 4°C. SYBR Premix Ex Taq II (Takara, Beijing, China) was used to detect cDNA expressions according to its protocols; the PCR cycling parameters are as follows: 95°C for 30 sec followed by 40 cycles at 95°C for 5 sec and 60°C for 30 sec. The relative expressions of various mRNA were normalized to *β*-actin or U6 by using 2^−△△CT^ method.

### 2.7. Protein Extraction and Western Blot

Total proteins of tissues and cells were extracted by using the protein extraction reagent (Beyotime, Shanghai, China) in line with its protocol. The concentrations were detected by using a BCA kit (Pierce Chemical Co., Rockford, IL, USA). 40 *μ*g total proteins were added onto the 10% SDS-PAGE for separation, which were transferred onto PVDF membranes. The PVDF membranes were blocked in the nonfatty milk at room temperature for 1 h and washed with TBST (Boster, China) for three times. Primary antibodies were obtained from Abcam (Abcam, Cambridge, USA). Cyclin D1 (ab16663, 1 : 200, 33 kDa), Cyclin E (ab33911, 1 : 1000, 47 kDa), N-cadherin (ab18203, 1 : 1000, 100 kDa), E-cadherin (ab40772, 1 : 10000, 110 kDa), Twist2 (ab66031, 1 : 1000, 18 kDa), and *β*-actin (ab8226, 1 : 5000, 42 kDa). PVDF membranes were, respectively, hatched with primary antibodies overnight at 4°C. After that, they were, respectively, hatched with the secondary antibody (1 : 5000) for another one hour. Proteins were detected in ECL detection system (Thermo Fisher Scientific, Shanghai, China).

### 2.8. CCK-8 Assay

Cell viability was detected by a cell counting kit-8 (CCK-8) assay (Dojindo, Rockville, Japan). Firstly, cells were prepared on 96-well plates (3 × 10^3^ cells/well) for 12 h, and three replicate wells were set for each group. And then, 10 *μ*l CCK-8 reagent was dripped into the prepared well in different time (24 h, 48 h, 72 h, and 96 h) and cultured for 2 h. Finally, the OD values of each well were detected at 450 nm by using a spectrophotometer (BioTek Instruments).

### 2.9. Transwell Assay

Cell migration was tested by the transwell assay. Firstly, target cells (1 × 10^4^ cells/well) were prepared into the upper Transwell chambers (BD Biosciences, NJ, USA) containing 10% FBS and 20% FBS was dripped to the lower chambers. Three replicate chambers were set for each experiment. After culturing for 24 h, the liquid in the upper chambers was removed and wished for three times, and the migrated cells were dripped with 95% methanol for 10 mins. Additionally, they were fixed with 0.5% crystal violet (Beyotime, Shanghai, China). Finally, the migrated cells were examined by using a light microscope (Olympus Corporation, Tokyo, Japan). Three independent experiments were repeated.

### 2.10. Luciferase Gene Reporter Assay

Dual-luciferase gene reporter assay was performed to confirm the direct relationship of circ_0067835 and miR-1236-3p and miR-1236-3p and Twist2. First of all, the wild and mutant sequences of circ_0067835 and Twist2 were, respectively, established and transfected into different GLO plasmids (Promega, USA). Then, HCC cells were, respectively, prepared in 48-well plates and cultured for 12 h. The two luciferase plasmids, including Renilla luciferase and firefly luciferase plasmids were transfected into the prepared cells for another 12 h. The indicated wild and mutant sequences were, respectively, transfected with Lipofectamine 2000 for 24 h. Additionally, miR-1236-3p mimics or mimics NC was, respectively, transfected into indicated cells for another 24 h. Finally, it was harvested, and luciferase activities were tested by using a luciferase assay system (Promega, USA).

### 2.11. Statistical Analysis

Data analysis was performed by using SPSS 22 and GraphPad Prism 6.0. Count data were processed by chi-square test, and the overall survivals of various HCC patient groups were analyzed by Kaplan-Meier survival test. Expression correlation analysis was performed by using Pearson's correlation method. Student's *t*-test or ANOVA was carried out to compare between various groups and SNK method was used for post hoc analysis. It was considered to be statistically different when *P* < 0.05.

## 3. Results

### 3.1. Circ_0067835 Was Elevated in HCC

In order to find out whether circRNAs showed different expression and had some functions in the development of human HCC, the microarray was performed with 3 paired tumor tissues and the adjacent normal tissues. The top 10 differentially expressed circRNAs were selected and the heatmap was displayed (Figure 1(a)), and circ_0067835 was obviously upregulated for about five folds in HCC tumor tissues. Then, 56 paired HCC tissues and adjacent normal tissues were used, and the expressions of circ_0067835 were tested with RT-PCR. It showed that circ_0067835 was obviously increased in HCC tumor tissues (*n* = 56) (Figure 1(b)). Furthermore, the levels of circ_0067835 in patients with metastasis (*n* = 29) were higher than those in patients without metastasis (*n* = 27) (Figure 1(c)). In addition, the levels of circ_0067835 in patients with larger tumor size (≥5 cm, *n* = 35) were higher than those in patients with smaller tumor size (<5 cm, *n* = 21) (Figure 1(d)). According to the expression of circ_0067835 in tumor, HCC patients were divided into the group of high circ_0067835 and low circ_0067835 by using the mean level of circ_ 0067835. Kaplan-Meier survival analysis indicated that the overall survival (OS) in HCC patients with circ_0067835 high expression group was lower than those in circ_0067835 low expression group (Figure 1(e)). And we detected the circ_0067835 expressions in various HCC cells, which showed that circ_0067835 were significantly increased in HCC cells (Figure 1(f)). Additionally, the clinicopathological analysis found out that the circ_0067835 level was extremely correlated to tumor size and distant metastasis in HCC patients (Table 1) (*p* < 0.05). As exhibited, circ_0067835 was upregulated in HCC.

### 3.2. Inhibition of Circ_0067835 Restrained the Capacities of Cell Proliferation and Migration in PLC5 and HepG2 Cells

Circ_0067835 si-RNA was constructed into a vector (si-circ_0067835) and were cotransfected into PLC5 and HepG2 cell lines, resulting with circ_0067835 inhibition (Figures 2(a) and 2(d)). CCK8 assays revealed that circ_0067835 inhibition significantly repressed cell viabilities after 72 h and 96 h (Figures 2(b) and 2(e)). Transwell assays indicated that inhibition of circ_0067835 obviously repressed cell migration in HCC cell lines (Figures 2(c), 2(f)). It had been widely accepted that Cyclin E and Cyclin D1 [25, 26] were associated with cell proliferation, N-cadherin, and E-cadherin were responsible for cell migration [9, 27]. WB assay revealed that the protein expressions of Cyclin D1, Cyclin E, and N-cadherin were reduced; E-cadherin protein expression was increased following with circ_0067835 inhibition in PLC5 and HepG2 cell lines (Figures 2(g)–2(i)).

### 3.3. miR-1236-3p Was Reduced in HCC Tissues, Which Was a Target of Circ_0067835 in PLC5 and HepG2 Cells

To investigate the regulatory mechanisms of circ_0067835 in HCC, the StarBase v2.0 was performed to find potential downstream miRNAs of circ_0067835. And we found 4 miRNAs were reported in other literatures among that, which were miR-377-5p, miR-324-5p, miR-545-3p, and miR-1236-3p, then we detected the expressions in tissue samples. No significant differences were found in miR-377-5p, miR-324-5p, and miR-545-3p (Figures 3(a)–3(c)), while miR-1236-3p was significant downexpressed in HCC samples (Figure 3(d)), which had been reported to regulate the development of various cancers [22–24, 28, 29], such as gastric cancer, lung cancer, colorectal cancer, prostate cancer, etc. Furthermore, miR-1236-3p in patients with metastasis was much lower than those without nonmetastasis (Figure 3(e)), and miR-1236-3p in patients with larger tumor size ( ≥5 cm, *n* = 35) was lower than those in patients with smaller tumor size (<5 cm, *n* = 21) (Figure 3(f)). Moreover, correlation analysis revealed that miR-1236-3p was negatively correlated with circ_0067835 in HCC patients with metastasis and larger tumor size (≥5 cm, *n* = 35) (Figures 3(g) and 3(h)). In addition, miR-1236-3p expressions were decreased in various kinds of HCC cells (Figure 3(i)), and it was increased following with circ_0067835 inhibition in PLC5 and HepG2 (Figure 3(j)). The wild type and mutant binding sequences of circ_0067835 were constructed and cotransfected into GLO vectors (Figure 3(k)). The luciferase gene reporter assays indicated that the activity was retrained after transfecting with WT-circ_0067835 and miR-1236-3p mimics, while no effects was found after transfecting with MUT-circ_0067835 and miR-1236-3p mimics in PLC5 and HepG2 cells (Figures 3(l) and 3(m)).

### 3.4. Upregulation of miR-1236-3p Could Restrain the Capacities of Proliferation and Migration in PLC5 and HepG2 Cells

miR-1236-3p mimics or mimics NC was, respectively, transfected into PLC5 and HepG2 cells, resulting with miR-1236-3p overexpression in both two cell lines (Figures 4(a) and 4(d)). Furthermore, CCK8 assays revealed that upregulation of miR-1236-3p could obviously restrain cell viabilities after 72 h and 96 h in PLC5 and HepG2 cells, compared with mimics NC groups (Figures 4(b) and 4(e)). Moreover, transwell assays indicated that upregulation of miR-1236-3p restrain migration capacity of PLC5 and HepG2 cells (Figures 4(c) and 4(f)). Besides, WB assay showed that upregulation of miR-1236-3p repressed the protein levels of Cyclin D1, Cyclin E, and N-cadherin, and accelerated E-cadherin in PLC5 and HepG2 cell lines (Figures 4(g)–4(i)).

### 3.5. The Elevated Twist2 Was a Direct Target of miR-1236-3p in PLC5 and HepG2 Cells

The Targetscan database and miRBase online were carried out to analyze the downstream targets of miR-1236-3p. Results showed that Twist2 had a high combining capacity according to the cumulative weighted combining score. Moreover, Twist2 had been showed to accelerate tumor progression, which was regarded as a poor diagnosis of HCC [30, 31], therefore, we tried to detect the expressions of Twist2 in HCC patients. Interestingly, western blot assay showed that the protein levels of Twist2 were significantly elevated in human HCC tumor tissues (Figure 5(a)). In addition, Twist2 protein levels in patients with metastasis and larger tumor size ( ≥5 cm, *n* = 35) were obviously higher than those patients with nonmetastasis and smaller tumor size (<5 cm, *n* = 21) (Figures 5(b) and 5(c)). Moreover, the protein levels of Twist2 were negatively correlated with miR-1236-3p in HCC patients with metastasis and larger tumor size ( ≥5 cm, *n* = 35) (Figures 5(d) and 5(e)). Additionally, Twist2 protein expressions were increased in HCC cells (Figure 5(f)), while they were repressed following with miR-1236-3p overexpression (Figures 5(g) and 5(h)). The wild type and mutant binding sequences for Twist2 were constructed and cotransfected into GLO vectors (Figure 5(i)). Luciferase gene reporter assays manifested that it was reduced after transfection with the WT-Twist2 and miR-1236-3p mimics, while it showed no difference after transfection with the MUT-Twist2 and miR-1236-3p mimics in both PLC5 and HepG2 cells (Figures 5(j) and 5(k)).

### 3.6. Circ_0067835 Accelerated Cell Proliferation and Migration through Interacting with miR-1236-3p/Twist2 Axis in Human HCC

In order to determine whether miR-1236-3p played critical roles in this axis, si-circ_0067835 was transfected into HCC cells, then miR-1236-3p inhibitor was also transfected to them. Results showed that the circ_0067835 was obviously restrained, and miR-1236-3p was escalated in si-circ_0067835 group, while circ_0067835 was escalated, and miR-1236-3p was restrained after cotransfecting with miR-1236-3p inhibitor in HCC cells (Figures 6(a) and 6(d)). Furthermore, CCK8 assays illustrated that the decreased cell viability in si-circ_0067835 was reversed after cotransfecting with miR-1236-3p inhibitor in HCC cells (Figures 6(b) and 6(e)). Besides, the transwell assays illustrated that the restrained cell migration capacity in si-circ_0067835 was reversed after cotransfecting with miR-1236-3p inhibitor HCC cells (Figures 6(c) and 6(f)). Additionally, WB assay revealed that the decreased protein levels of Twist2, Cyclin D1, Cyclin E, and N-cadherin in si-circ_0067835 were increased following with miR-1236-3p inhibitor transfection, while the accelerated E-cadherin in si-circ_0067835 was decreased after cotransfecting with miR-1236-3p inhibitor (Figures 6(g)–6(i)).

## 4. Discussion

HCC is one of the leading causes of human cancer-related death around world. HCC patients at advanced stages show a poor prognosis with a mean survival date, and patients with advanced HCC have little treatments [2–5]. Therefore, we should find new diagnostic markers to make earlier diagnoses and identify therapeutic targets to improve the clinical efficacy for HCC patients. circRNAs have been revealed to regulate cancer cell biological functions through the ceRNA mechanism in HCC [10–12, 32–35]. More investigations on the mechanisms of underlying HCC cell proliferation and metastasis are of great significant.

Circ_0067835 was demonstrated to accelerate the malignant progression of endometrial cancer cells through modulating miR-545-3p/FAM98A signaling pathway [14]. It had been revealed that circ_0067835 knockdown could suppress cell progression and enhance cell radiosensitivity of colorectal cancer partially by sponging with miR-296-5p/IGF1R axis [15]. But the roles of it in HCC remained unclear. Therefore, the microarray and other experiments were performed. Current results illustrated that circ_0067835 was obviously escalated in HCC. It was a topic of interest, which was related to tumor size and metastasis in HCC patients.

To investigate the functions of circ_0067835 in HCC, si-circ_0067835 was constructed and cotransfected into HCC cells to inhibit circ_0067835 expression. Results indicated that circ_0067835 inhibition repressed cell proliferation and cell migration in HCC cells. Cyclin D1 and Cyclin E are critical proteins that are responsible for cell proliferation in various cancers [25, 26]. N-cadherin is responsible for promoting cell invasion and migration, while E-cadherin is responsible to inhibit cell invasion and migration [9, 27]. WB assay demonstrated that circ_0067835 inhibition decreased the levels of Cyclin D1, Cyclin E, N-cadherin, and increased E-cadherin, which confirmed that circ_0067835 inhibition repressed cell proliferation and cell migration. However, the mechanism remained unknown.

It has been widely revealed that circRNAs are of vital importance in biological functions of various cancers through interacting with miRNAs, which can serve as ceRNAs [10–12]. For example, the upregulated circ_001306 could enhance cell proliferation of HCC through interacting with miR-584-5p/CDK16 signaling pathway [10]. Therefore, we analyzed the potential downstream miRNAs of circ_0067835, which illustrated that miR-1236-3p might be one of them. Current results manifested that miR-1236-3p levels were reduced in HCC patients that were negatively correlated with circ_0067835. And it had been verified by luciferase reporter assay in HCC cells. Recent evidence manifested that miR-1236-3p was involved in some digestive system cancers, such as gastric cancer [22, 23] and colorectal cancer [24], but the roles in HCC were little known. And current results illustrated that upregulation of miR-1236-3p could obviously restrain capacities of cell proliferation and migration. It has also been demonstrated that miRNAs can affect various cell functions by directly binding with the 3′-UTR of downstream target genes in diseases [36, 37], including HCC [38–40]. Then, the potential target genes of it were performed by utilizing the Targetscan database and miRBase.

Twist2 has been demonstrated to be an important regulator and a poor diagnosis marker in some cancers [41–44], such as gastric cancer [42], cholangiocarcinoma [41], glioma [43], etc. Importantly, it has been revealed that it could accelerate cell proliferation, metastasis, and epithelial-mesenchymal transition (EMT) in HCC [30, 31, 45]. And the Twist2 protein levels were obviously increased in HCC tumor tissues, which were negatively related to miR-1236-3p, while it was positively related to circ_0067835. And our assumption was certificated by luciferase reporter assay in HCC cells. Finally, the miR-1236-3p inhibitor was used to observe whether it could reverse the effects after transfecting with circ_0067835. Current results showed that the strained capacities of proliferation and migration in HCC cells were ameliorated, which suggested that circ_0067835 could accelerate these capacities through interacting with miR-1236-3p/twist2 axis in HCC patients.

In this study, we found that circ_0067835 was ameliorated in HCC, which was a prognostic marker for HCC patients. Additionally, we illustrated that circ_0067835 could accelerate proliferation and migration of HCC cells. Surprisingly, results demonstrated that the elevated circ_0067835 could directly interact with miR-1236-3p. It could increase twist2 expression, which could accelerate cell proliferation and metastasis in HCC. We uncovered a circle RNA that might predict the prognosis for HCC patients, which provided a new insight for treating HCC.

## 5. Conclusion

To conclude, we found out that circ_0067835 was elevated in HCC, which could accelerate capacities of proliferation and migration through interacting with miR-1236-3p and accelerating Twist2 in HCC. Loss of it could significantly inhibit the progression of HCC, which provided a novel therapeutic target for HCC patients.

## Figures and Tables

**Figure 1:** Circ_0067835 was elevated in HCC. (a) Microarray was performed with 3 paired tumor tissues and adjacent nontumor tissues of HCC patients, and top 10 differentially expressed circRNAs were displayed in the heatmap. (b) RT-PCR was carried out to test circ_0067835 in HCC tumor (*n* = 56) and adjacent nontumor tissues (*n* = 56). (c) Circ_0067835 expressions in HCC patients with metastasis (*n* = 29) and nonmetastasis (*n* = 27). (d) Circ_0067835 expressions in HCC patients with larger tumor size ( ≥5 cm, *n* = 35) and smaller tumor size ( <5 cm, *n* = 21). (e) Kaplan-Meier survival analysis was performed to analyze the overall survival rates for low and high circ_0067835 expression patients. (f) RT-PCR was utilized to test circ_0067835 levels in HCC cells. ^∗^*p* < 0.05, ^∗∗^*p* < 0.01, and ^∗∗∗^*p* < 0.001.

**Figure 2:** Inhibition of circ_0067835 restrained the capacities of cell proliferation and migration in PLC5 and HepG2 cells. Si-circ_0067835 or si-NC was constructed into the vectors and transfected into HCC cells. (a and d) Circ_0067835 expressions were detected after transfection by RT-PCR. (b and e) Cell viabilities were measured by CCK8 assay. (c and f) Transwell assays (Magnification, x100) were carried out to test cell migration capacity. (g–i) Protein expressions of Cyclin D1, Cyclin E, N-cadherin, and E-cadherin were detected by WB assay (magnifications x 1.0). ^∗∗^*p* < 0.01 and ^∗∗∗^*p* < 0.001.

**Figure 3:** miR-1236-3p was reduced in HCC tissues, which was a target of circ_0067835 in PLC5 and HepG2 cells. (a–d) RT-PCR was performed to detect several miRNA levels in HCC tumor (*n* = 56) and nontumor tissues (*n* = 56). (E) miR-1236-3p expressions in HCC patients with metastasis (*n* = 29) and nonmetastasis (*n* = 27). (f) miR-1236-3p expressions in HCC patients with larger tumor size ( ≥5 cm, *n* = 35) and smaller tumor size ( <5 cm, *n* = 21). (g and h) Correlation analysis was performed between circ_0067835 and miR-1236-3p in patients with metastasis and larger tumor size (≥5 cm, *n* = 35). (i and j) miR-1236-3p expressions were detected in HCC cells and in HCC cells after transfection with si-NC or si-circ_0067835. (k) Wild type and mutant binding sequences of circ_0067835 were constructed and cotransfected into GLO vectors. (l and m) Luciferase gene reporter assay was performed in HCC cells. ^∗∗^*p* < 0.01 and ^∗∗∗^*p* < 0.001.

**Figure 4:** Upregulation of miR-1236-3p could restrain the capacities of proliferation and migration in PLC5 and HepG2 cells. (a and d) miR-1236-3p expressions were tested by RT-PCR. (b and e) Cell viabilities were measured by CCK8 assay. (c and f) Cell migration capacity was measured by transwell assay (Magnification, ×100). (g–i) Protein expressions of Cyclin D1, Cyclin E, N-cadherin, and E-cadherin were detected by WB assay (magnifications × 1.0). ^∗∗^*p* < 0.01 and ^∗∗∗^*p* < 0.001.

**Figure 5:** The elevated Twist2 was a direct target of miR-1236-3p in PLC5 and HepG2 cells. (a) WB assay was carried out to test Twist2 in HCC tumor (*n* = 56) and nontumor tissues (*n* = 56). (b) Twist2 protein levels in HCC patients with metastasis (*n* = 29) and nonmetastasis (*n* = 27). (c) Twist2 protein levels in HCC patients with larger tumor size ( ≥5 cm, *n* = 35) and smaller tumor size ( <5 cm, *n* = 21). (d and e) Correlation analysis was performed between Twist2 and miR-1236-3p in patients with metastasis and larger tumor size ( ≥5 cm, *n* = 35). (f) Twist2 protein expressions were tested in HCC cells and in HCC cells. (g and h) Twist2 protein levels were detected in PLC5 and HepG2 cells after transfecting with mimics NC or miR-1236-3p mimics. (i) Wild and mutant sequences of Twist2 were constructed and cotransfected into GLO vectors. (j and k) Luciferase gene reporter assay was carried out in PLC5 and HepG2 cells. ^∗^*p* < 0.05, ^∗∗^*p* < 0.01, and ^∗∗∗^*p* < 0.001.

**Figure 6:** Circ_0067835 accelerated cell proliferation and migration through interacting with miR-1236-3p/Twist2 axis in human HCC. (a and d) Circ_0067835 and miR-1236-3p expressions were tested by RT-PCR in PLC5 and HepG2 cells. (b and e) Cell viabilities were measured by CCK8 assay. (c and f) Cell migration capacities were measured by transwell assay (Magnification, ×100). (g–i) Protein expressions of Cyclin D1, Cyclin E, N-cadherin, and E-cadherin were detected by WB assay (magnifications × 1.0). ^∗∗^*p* < 0.01, and ^∗∗∗^*p* < 0.001.

**Table 1:** Correlation between circ_0067835 level and clinicopathological features in HCC patients.

Parameters	Total patients (*n* = 56)	Low circ_0067835 expression (*n* = 28)	High circ_0067835 expression (*n* = 28)	*P* value
Age				0.781
<65Y	26	17	9	
≥65Y	30	11	19	
Gender				0.391
Male	38	21	17	
Female	18	7	11	
Tumor size				
<5 cm	21	15	6	0.026^∗^
≥5 cm	35	13	22	
TNM stage				
I-II	26	17	9	0.059
III-IV	30	11	19	
Metastasis				
Yes	29	9	20	0.007^∗^
No	27	19	8	

**Table 2:** Primer sequences for RT-PCR.

Gene names	Primer sequences	Species
circ_0056618	Forward: 5′- GAACCCACCCCACCTCTAC-3′	Human
	Reverse: 5′-CTTCCCCGGGATAAACAAACC-3′	
miR-1236-3p	Forward: 5′- AACAAGCCTCTTCCCCTTGT-3′	Human
	Reverse: 5′- GTCGTATCCAGTGCAGGGT-3′	
miR-377-5p	Forward: 5′-CAGGUCACGUCUCUGCAGUUAC-3′	Human
	Reverse: 5′- GTGCGTGTCGTGGAGTCG-3′	
miR-324-5p	Forward: 5′- GCTATCACAGAGCATTTTCTCAT-3′	Human
	Reverse: 5′- TGCACCAAACACGACTTTTAACC -3′	
miR-545-3p	Forward: 5′-TGG CTC AGT TCA GCA GGA AC-3′	Human
	Reverse: 5′- TGG TGT CGT GGA GTCG-3′	
*β*-actin	Forward:5′-GCTTCGGCAGCACATATACTAAAAT-3′	Human
	Reverse:5′-AGGGTACATGGTGGTGCCGCCA-3′	
U6	Forward:5′-CGCTTCACGAATTTGCGTGTC-3′	Human
	Forward:5′-TAAAACGCAGCTCAGTAACAGTC-3′	

## Data Availability

Citations should appear in the body of the article with a corresponding reference in the reference list.
